# A Novel Bitcoin and Gold Prices Prediction Method Using an LSTM-P Neural Network Model

**DOI:** 10.1155/2022/1643413

**Published:** 2022-05-05

**Authors:** Xinchen Zhang, Linghao Zhang, Qincheng Zhou, Xu Jin

**Affiliations:** ^1^School of Telecommunications and Information Engineering, Nanjing University of Posts and Tele-Communications, Nanjing 210046, China; ^2^School of Science, Nanjing University of Posts and Telecommunications, Nanjing 210046, China

## Abstract

As a result of the fast growth of financial technology and artificial intelligence around the world, quantitative algorithms are now being employed in many classic futures and stock trading, as well as hot digital currency trades, among other applications today. Using the historical price series of Bitcoin and gold from 9/11/2016 to 9/10/2021, we investigate an LSTM-P neural network model for predicting the values of Bitcoin and gold in this research. We first employ a noise reduction approach based on the wavelet transform to smooth the fluctuations of the price data, which has been shown to increase the accuracy of subsequent predictions. Second, we apply a wavelet transform to diminish the influence of high-frequency noise components on prices. Third, in the price prediction model, we develop an optimized LSTM prediction model (LSPM-P) and train it using historical price data for gold and Bitcoin to make accurate predictions. As a consequence of our model, we have a high degree of accuracy when projecting future pricing. In addition, our LSTM-P model outperforms both the conventional LSTM models and other time series forecasting models in terms of accuracy and precision.

## 1. Introduction

The financial markets have a magical air that attracts a varied spectrum of investors to take part in the game of chance. In recent years, the rapid rise of financial technology and artificial intelligence has led to their widespread use across a broad range of sectors, including methods such as machine learning and deep learning, among others. When it comes to the interpretation and prediction of temporal data, deep learning algorithms have made significant strides. The use of quantitative algorithms is becoming more popular in conventional financial markets, such as futures trading and stock trading, as well as in other financial markets, such as digital currency exchanges. It is the systematic process of executing automated preprogrammed trading instructions while accounting for factors such as volume, price, and time in order to maximize profit and minimize risk. When it comes to trading in the financial market, it employs complex mathematical algorithms to increase the efficiency of trading choices. As a result of using sophisticated algorithms in combination with mathematical models and human supervision, it makes trading decisions on exchanges. Furthermore, according to the Financial Times, quantitative trading is increasingly being utilized to trade digital currencies (e.g., Bitcoin) in addition to the traditional hedge fund and futures trading. Numerous quantitative strategies have benefitted from the high volatility of digital currencies, which has resulted in an increase in the rate of return. In general, we believe that a quantitative strategy involves a thorough examination of market characteristics, market sentiment, and other varied information in order to obtain maximum returns with relatively tolerable risk. Based on research, according to the study, the Algorithmic Trading Market was valued at USD 11.66 billion in 2020 and is predicted to expand to USD 26.27 billion by 2028, growing at a compound annual growth rate (CAGR) of 10.7 percent between 2021 and 2028.

According to our beliefs, the price movement of an investment is the consequence of a dynamic game in which a number of different people participate, and we think that although the market is nonlinear, there are some patterns that may be seen. We might infer from the principles that underpin technical analysis that history is a repeating cycle. Numerous time series of the financial market have been discovered to include stylized facts of the financial market, and there are many stylized facts of financial market indexes to be found [1, 2] as well. As a result, in this paper, we will discuss ways for forecasting market prices.

The time series analysis method is one of the quantitative forecasting approaches that are now accessible on the market. The creation and inference of statistical models, as well as the most optimal time series prediction, control, and filtering, are all discussed in detail. Time series analysis may be separated into two forms: deterministic change analysis and random change analysis. Deterministic change analysis is the more common of the two types. Trend change analysis, cycle change analysis, and random change analysis are all types of deterministic change analysis, while random change analysis includes AR, MA, and the ARMA model. Some forms of random change analysis are covered in this section of the manual.

Traditionally used time series forecasting models, such as the ARIMA [3] and Vector Autoregressive Model (VAR) [4], have some drawbacks due to the fact that the investment market is a nonlinear nonhomogeneous system. Machine learning, on the other hand, thanks to its improved performance, can carry out efficient excavation in order to get prospective information from the market. In recent years, the application of machine learning in market forecasting has grown in importance, and it has largely exceeded the prediction accuracy of classical time series forecasting models in terms of accuracy.

Price prediction models based on neural networks, such as recurrent neural networks (RNN) [5], convolutional neural networks (CNN), multilayer perceptron (MLP) [6, 7], and long short-term memory (LSTM) [8], have proven to be the most widely used among machine learning approaches in recent years. For the period between March 11, 2014, and March 31, 2019, Soylemez used a multilayer artificial neural network technique to estimate gold prices, utilizing parameters such as Brent oil prices, the VIX index, the Dow Jones index, and the US Dollar index [9]. In order to forecast the stock prices of selected companies, a long short-term memory model is utilized to analyze the daily stock price movement and returns of different sectors based on their prior values [10]. Using a DAE LSTM model [11], Sanghyuk's study suggests that the proposed approach may be used to predict future stock prices. A short-term memory network (LSTM) on the basis of a convolutional neural network has been added to considerably improve the prediction capacity of gold volatility. However, despite the fact that deep learning has shown substantial success in time series prediction, particularly in the financial industry, building and selecting the best-suited strategy for a researcher is a time-consuming and challenging procedure.

Due to the fact that prices are impacted by a wide range of macro- and microeconomic variables (for example, investor attitude), price changes may be quite severe. The process of dramatic fluctuations generates a huge quantity of noisy data, which is also created throughout the process. As a result, when a single machine learning model is used to anticipate prices, there is a significant amount of prediction error. As a result, we wish to increase the accuracy of predictions by the combined usage and refinement of models, as well as by introducing some novel concepts (e.g., LSTM-P).

The following are the particular contributions that we have made:

1. Achieve noise reduction by the application of the wavelet transform: this paper presents a novel noise reduction strategy based on the wavelet transform that is used to smooth the fluctuations of price data and increase the accuracy of future forecasts in order to reduce the impact of high-frequency noise components on pricing.
2. Develop an LSTM prediction model that is as accurate as possible (LSPM-P): to anticipate future gold and Bitcoin prices, we create an upgraded LSTM prediction model (LSPM-P) and train it using past gold and Bitcoin price data. This is the second stage. If we look at the conclusion of our model, we can see that it has a high degree of accuracy when it comes to anticipating future prices. As previously stated, our LSTM-P model outperformed both conventional and other time series forecasting models in terms of accuracy and precision, as well as other time series forecasting models.

## 2. Related Works

### 2.1. Long Short-Term Memory

It was Hochreiter and Schmidhuber who first proposed the long short-term memory (LSTM) neural network in 1997, and it has subsequently gained widespread acceptance. Afterwards, it was fine-tuned over a period of many years. Since the introduction of the “gate” component into the LSTM framework, it has become more popular. Using the “gate” structure, it is possible to choose the most effective feature for processing from a huge number of characteristics and achieve the aim of controlling the flow of information [12]. LSTM neural networks include numerous neurons called storage units in the hidden layer, and each storage unit has three “gates.” This class of “gates” is referred to as forgetting gates (*f*_*t*_), input gates (*i*_*t*_), and output gates (*o*_*t*_). One of the capabilities of an LSTM neural network is the ability to control the transmission of input data; additionally, the independence between the memory storage unit output and result output can be maintained, allowing the sequence to retain important information during transmission as well as the ability to retain longer-term memories, among other things. Thus, it is advised that the LSTM neural network can be used for time series prediction in the financial industry.

The following sections detail the processes involved in training an LSTM neural network. First, we can figure out what the network topology and loss function of the LSTM are. Second, initialize each parameter, and then, using the loss function, determine the accuracy rate of the model as a percentage. If it is unable to achieve the required precision, we will need to make changes to the settings. The weight and the size condition for updating bias terms should be that they minimize the loss of the stated objective function in the training sample, which is referred to as the pass loss in the training sample. When comparing and contrasting parameters, the function collects the gradient information, which is subsequently used to update parameters in accordance with the model's learning rate. As a general rule, we shall choose the most appropriate optimization procedure to update the gradient value. Consequently, when the gradient achieves the needed accuracy, the parameters of the model can be computed, the LSTM model can be finished, and the model may be used for prediction or classification.

Because of its memory units and “gates,” the LSTM is capable of dealing with issues that the RNN was unable to handle. It can also carry out long-term memory storage of essential information in a quick and efficient way, and it can learn successfully via these mechanisms. As a consequence, a substantial amount of research has been conducted on financial time series modeling as a result of these developments. In spite of the fact that the neural network's revenue distribution closely mirrored that of Bitcoin, Wang et al. concluded that more advanced learning algorithms such as deep cyclic neural networks, RNN, and LSTM may give superior forecast accuracy [13]. When estimating Bitcoin, Wu et al. compared the ARIMA time series model with the LSTM deep learning model, which she found to be superior. As a result, the average absolute error of the LSTM model was much lower than that of the ARIMA model. The results show that the LSTM model was significantly accurate in forecasting the price of special currency [14]. The sophisticated temporal aspects of machine learning methodologies led Marendra et al. to discover that cyclic neural networks and long short-term memory neural networks were more accurate at forecasting Bitcoin prices than traditional multilayer perceptron (MLP) neural networks [15, 16]. This study is built on an LSTM network as a basis, since it is effective at learning the correlation of time in a sequence and has a broad variety of applications in the field of time series prediction.

### 2.2. Attention Mechanism

The amount of information that a neural network is capable of storing is referred to as the network capacity of the particular neural network under consideration. The increase of the number of neurons in the network will lead to the corresponding increase in network capacity. Because the capacity of a network increases with its size, the number of neurons increases as well, making the network more complex overall. As a consequence, the bigger the number of parameters in the neural network, the more complex the network. It is not suggested to increase the complexity of the model to improve its expressiveness due to the limitations in the processing capability of the computer. The outcome has been the development of an attention mechanism that is inspired by the mechanics of the human brain, which may be used to cope with the challenges associated with information overload. It is no longer necessary for the attention mechanism to pay attention to data characteristics from all areas; instead, it only needs to pay attention to data characteristics from critical locations, resulting in significant time savings. In addition to saving a substantial amount of time by removing an enormous number of pointless calculations, this may improve the accuracy and generalization of the model by increasing its generalization and accuracy [17].

According to the attention mechanism, data with dynamic change characteristics may be captured more efficiently, resulting in a more accurate correlation analysis. It is suggested that the attention method should be introduced into the prediction of time series data prediction. Wang et al. used the LSTM model, which is based on attention, to forecast the day when the SSE 50 daily closing price will be reached. In this study, he looked at a single-factor LSTM model that did not include the attention mechanism and contrasted it with the conventional LSTM model. Aside from that, he looked at two other versions of the attention mechanism, one with and one without the decoding process, and he compared them to one another. Although the attention-LSTM model without the decoding process trained more quickly than the model with the decoding process, the prediction accuracy of the model without the decoding process was not as good as that of the model with the decoding process [18]. Wang et al. proposed a random recursive network called the CLVSA model. Researchers claim that their technique may be used to predict likely variations in raw financial transaction data. Based on deep LSTM and attention mechanisms, Zheng and Xu have developed a financial data forecasting strategy that is based on deep LSTM and attention mechanisms [19]. This study used daily data as well as time-sharing data to investigate the influence of capital flow variations on stock trend changes, with the finding that the self-attention model is enhanced as a consequence. As a result of the experiments, the suggested technique was able to improve the accuracy of trend judgment to 63.04 percent and gain 6.562 percent in the two-month backtest experiment, demonstrating that the model has a certain level of efficacy and practicability in the prediction of stock price trends. LSTM has encountered a number of obstacles in the area of financial time series prediction. Improving the LSTM model is essential for producing more accurate results in the highly dynamic field of investment forecasting. According to the article, this model is referred to as the LSTM-P model.

## 3. Bitcoin and Gold Prices Prediction

### 3.1. Data

The data employed in our model for the empirical application consist only of historical price series for Bitcoin and gold, which were collected between September 2016 and September 2021. Gold daily prices (in US dollars per troy ounce) are sourced from the London Bullion Market Association, while Bitcoin daily prices (in US dollars per Bitcoin) are sourced from the Nasdaq Stock Market. Take a look at Figures 1 and 2.

Note: Bitcoin can be traded every day, so the data are continuous. However, gold has a difference between trading days and nontrading days and the data are not continuous. We first do a smoothed interpolation of the historical price of gold to facilitate the forecasting model. Moreover, we consider the nontrading day scenario in the trading strategy.

### 3.2. Flow of Our Work

Considering the background information and restricted conditions, the article consists of three parts. The first one is data preprocessing part. We use interpolation fitting and wavelet transform noise reduction for Bitcoin and gold historical price data, in order to get higher accuracy in the later time series prediction. Then, we use a modified LSTM-Plus (LSTM-P) neural network for training and prediction. LSTM-P is characterized by keeping only one control gate in the original LSTM model and adding cellular connections to the candidate hidden states and control gate to improve prediction accuracy. At last, we make a sensitivity analysis. In order to avoid complicated descriptions and intuitively reflect our work process, the specific flowchart of the full article can be referred to in Figure 3.

For the purposes of this work, Python 3.8 is used for data preparation and processing, with the programs NumPy, TensorFlow, and Keras serving as support. These tools are used to complete the model construction process. In addition, we utilize SPSS25 to evaluate the data.

### 3.3. Model Preparation

#### 3.3.1. General Assumptions and Justifications

To make the issue easier to understand, we make the following fundamental assumptions, each of which is supported by appropriate evidence.

**Assumption 1 .**

Prices reflect all information.

Justification: this is the basic principle of technical analysis. Whether it is fundamental information or investor behavior and sentiment, it is ultimately reflected in price changes. Investors' reasons and thinking for making trading strategies are like the hidden layer of a neural network. Thus, we have no need to overthink and we just need to know the results, which is one of the reasons why we choose a neural network to forecast.

**Assumption 2 .**

We do not consider high-frequency trading and shorting trading.

Justification: there are high transaction costs, and we only have daily price data, so we only consider swing trading and the trading frequency will not be too large. Moreover, there is no shorting mechanism, only spot buy and sell operations are allowed.

#### 3.3.2. Data Noise Reduction

Bitcoin and gold price data are trend-like time series data, and we usually differentiate the data first. However, because of various factors, the volatility of gold and Bitcoin prices is very sharp (e.g., Bitcoin), leading to large price fluctuations in the short term and generating a lot of white noise. Therefore, the different methods will not be good for the trend prediction results. We need to perform volatility smoothing on the time series of prices to some extent, so that the trending characteristics can be retained and the noise is reduced.

If you are looking for a method that can be used for time-frequency analysis, wavelet analysis is one that you should consider. Data scaling and panning are used in this method; as a result, it is capable of examining both time-domain and frequency-domain components of a signal at the same time. The wavelet technique [6] may be used to split a noisy signal into numerous scales and denoise the signal while keeping its integrity. This is true regardless of the frequency content of the signal. As a result of its adaptive characteristics, wavelet analysis is particularly well suited for problem signals that are smooth and nonlinear in nature. Liu et al. used the wavelet transform to their data in order to reduce the amount of noisy data they had. Mallick et al. proposed a novel approach for increasing the prediction accuracy of noisy multivariate time series that are based on the wavelet-denoising algorithm and multiple echo state networks. When it comes to precision, it exceeds both the Fourier transform and the window Fourier transform together.

If a time series function *f*(*t*) ∈ *L*^2^(*R*) and when the following conditions are met,

(1) $$\begin{array}{c} C_{W}=\int_{0}^{\infty }\frac{{\left|\psi \left(\omega \right)\right|}^{2}}{\omega }\text{d}\omega <\infty , \end{array}$$

where *ψ*(*t*) is the mother wavelet function and *ψ*(*ω*) is the Fourier transform of the mother wavelet function, then we can get

(2) $$\begin{array}{c} W\left(a,\tau \right)=\int_{-\infty }^{+\infty }f\left(t\right){\bar{\psi }}_{a,\tau }\left(t\right)\text{d}t,\\ f\left(t\right)=\frac{1}{C_{\psi }}\int_{-\infty }^{+\infty }a^{-2}W\left(a,\tau \right)\psi_{a,\tau }\left(t\right)\text{d}a\text{d}\tau , \end{array}$$

where the displacement and scaling of the fundamental wavelet is

(3) $$\begin{array}{c} \psi_{a,\tau }\left(t\right)=\frac{1}{\sqrt{a}}\psi \left(\frac{t-\tau }{a}\right), \end{array}$$

where *a* is the scale factor, *τ* is the translation variable, and equation (3) is the continuous wavelet transform. Next, the signal is decomposed (equation (4)) and reconstructed (equation (5)):

(4) $$\begin{array}{c} c_{k}^{j}=\sum_{n}H\left(n-2k\right)c_{n}^{j-1}, \end{array}$$

(5) $$\begin{array}{c} c_{n}^{j-1}=\sum_{n}h\left(n-2k\right)c_{k}^{j}+\sum_{n}g\left(n-2k\right)d_{k}^{j}. \end{array}$$

The low-pass filter is *H*(*n*), and the low-pass impulse response is *h*(*n*). The high-pass filter is *G*(*n*), and the high-pass impulse response is *g*(*n*). The low-frequency signal is *c*_*k*_^*j*^, which contains less noise, and the high-frequency signal is *d*_*k*_^*j*^, which has more noise.

Because the deconstructed high-frequency data include practically all of the noise, the high-frequency signal must first be denoised according to the threshold value and then the low-frequency and denoised high-frequency sections must be rebuilt from the low-frequency data.

The reconstructed data are the denoised data, which finally complete the whole denoising process.  Figure 4 shows the whole process (taking 2-layer decomposition as an example).

On the basis of the foregoing, it can be concluded that, because the trending characteristics of the low-frequency part of the price time series data are the most important information, it is possible to remove noise from the data by performing noise reduction on the price time series data in order to improve the accuracy of prediction by the neural network model by using neural networks.

#### 3.3.3. Data Analysis after Preprocessing

We choose db8 wavelets in the original signal decomposition process and performed a 6-layer decomposition of the signal. The figures below show the data after noise reduction by wavelet transformation (using Bitcoin as an example). We find that the processed data have a smoothing effect in time regions with high short-term fluctuations. Small fluctuations have been largely eliminated and almost no longer contain noisy data.  Figure 5 shows the comparison of data before and after processing in a time region with high Bitcoin fluctuations.  Figure 6 shows a before-and-after comparison of all Bitcoin data.

The error rates before and after data processing are shown in Figure 7.

Taking Bitcoin as an example, we find that the average error rate of the data after noise reduction by wavelet transform is 0.03. We then differentiate the data before and after processing to get the increase and decrease of each day relative to the previous day. Calculating their statistical features (Table 1), we find that the variance of the processed data is much lower, achieving the effect of smoothing fluctuations. In addition, the larger the value of the signal-to-noise ratio (SNR), the smaller the noise of the data after noise reduction, and the smaller RMSE indicates that the noise reduction process changes the trend of the original data less.

### 3.4. Time Series Prediction (LSTM-P)

#### 3.4.1. Description of the Model

When it comes to time series prediction, it is widely accepted that LSTM (long short-term memory) neural networks do very well in this area. A higher memory function than other creatures may be found in its cell structure. LSTM networks filter input in order to maintain and update the state of storage cells. This is accomplished via the use of gating mechanisms. Gating in the model may be divided into three types: in-going gates, forgetting gates, and output gates. The storage cell has three sigmoid layers and one tanh layer, and the model also has three sigmoid layers and one tanh layer, with three sigmoid levels and one tanh layer. LSTM storage cells are shown in Figure 8 as having a common structural layout.

LSTM models are very advanced when it comes to time series prediction, but they still have a number of shortcomings that must be addressed. The training efficiency and prediction accuracy of a model will both suffer if the number of layers in the model is excessive, as in the case of a multilayer model. Because of this, we are striving to strengthen the existing model by adding both the mature model and some other superior models [20, 21], which may not only simplify the model but also increase prediction accuracy as a result of the improved models.

We create a new LSTM model called LSTM-Plus (LSTM-P), which has been proven to improve the prediction accuracy. LSTM-P has the following features:

- Coupled input gate and forgetting gate.
- The previous moment cell state is added to the gating of the coupled input and forgetting gates. That is, the more important part of the model is the candidate's hidden state of the previous moment, which allows the gating to more accurately select the information that needs to be input versus forgotten.
- A constant column vector *β* is subtracted before the coupled gating activation (the value of *β* depends on the predicted dataset, usually set to 1). This will allow accumulating slightly more information than the amount of information forgotten, making it easier to analyze the time series.

Figure 9 depicts the structure of the enhanced LSTM-P model.

The neurons of the improved LSTM-P model are specifically interpreted as follows:

(6) $$\begin{array}{c} f_{t}=\left(W_{f}\left[c_{t-1},h_{t-1},x_{t}\right]+b_{f}\right),\\ \tilde{C}=\tanh\left(W_{c}\left[h_{t-1},x_{t}\right]+b_{c}\right),\\ C_{t}=\sigma \left(f_{t}\right)*C_{t-1}+\left(1-\sigma \left(f_{t}-\beta \right)\right)*{\tilde{C}}_{t},\\ h_{t}=C_{t}. \end{array}$$

#### 3.4.2. Training of Our Model

We train the Bitcoin and gold price data separately and do incremental training on each other. We divide the dataset in a 4 : 1 ratio, with a total of 1826 pieces of data. We use the first 50 days of prices to predict the last 5 days of prices. After determining the input data for the model, we train and predict a 2-layer LSTM-P model.

Several parameters were changed during the process, such as the epoch used to compare the loss function and the value of the overfitting dropout function. In addition, we do a comparison between the LSTM-P model and the LSTM model prediction results.

For our final fixed epoch is equal to 30, as shown in Figure 10, the loss function is less than 0.05 and the final MAPE is less than 0.05.

In addition, the comparison shows that the LSTM-P model we use has a faster convergence rate of the decreasing loss function than the general LSTM model. When the dataset is not denormalized, the value of the loss function (MAPE) of our LSTM-P model is 0.0481 after 30 training sessions, which is better than that of the LSTM at 0.0608 (Table 2).

#### 3.4.3. Results of Our Model

Figures 11 and 12 show the predicted data for Bitcoin and gold prices compared to the source data. We define an indicator error rate (ER, equation (7)) to compare the degree of error of the predicted data to the original data.

(7) $$\begin{array}{c} \text{ER}=\;\frac{\left(\text{value}-\text{metavalue}\right)}{\text{metavalue}}. \end{array}$$

We calculate the error rate and depict it with scatter plots in Figures 11 and 12.

Figures 13 and 14 show the forecast data for Bitcoin and gold for some time periods.

Based on the error rate analysis and the results of prediction above, we conclude that our prediction model is valid. We find the following conclusions:

- The average error rate for gold price prediction is 0.0094, which is smaller than Bitcoin's 0.0382.
- Note: this is also in line with common sense. As Bitcoin's volatility is much greater than that of gold, even after our wavelet noise reduction, Bitcoin's price prediction still has more errors than gold's.
- Because of the limited amount of data available before training, the estimates for the two underlying investments exhibit large errors in the first few hundred days.
- We backtest some of the time periods with large errors (i.e., time periods with large price swings). These periods tend to have prices that are out of character with previous movements of this investment variety.
- Note: we feel that perhaps this is because of the excessive irrational emotional manipulation of investors at this time, causing large ups and downs. It is like a sudden change in a person's personality. These are the times when forecasting models are of little use.

## 4. Conclusions

The trained LSTM-P model predicts BTC and gold data with a somewhat high degree of accuracy for both BTC and gold. Several times during the training process, we made adjustments to the parameters (epoch, layer, and so on) in order to get a prediction model that was close to ideal. When compared to the general LSTM model, our model has been significantly optimized (explained above). If more optimization is required, the inclusion of an attention layer may be explored.

## Figures and Tables

**Figure 1:** Gold daily price.

**Figure 2:** BTC daily price.

**Figure 3:** Flowchart of our work.

**Figure 4:** Two-layer wavelet noise reduction schematic.

**Figure 5:** BTC before and after noise reduction. (a) Example of data before noise reduction. (b) Example of data after noise reduction.

**Figure 6:** BTC before and after noise reduction.

**Figure 7:** Error rate of prices data.

**Figure 8:** Structure of a typical LSTM storage cell.

**Figure 9:** Structure of the LSTM-P model.

**Figure 10:** Train loss charts.

**Figure 11:** Error rate scatter plot by BTC forecast price vs. metadata.

**Figure 12:** Error rate scatter plot by gold forecast price vs. metadata.

**Figure 13:** Forecast data for Bitcoin.

**Figure 14:** Forecast data for gold.

**Table 1:** Statistical characteristics of the data before and after processing.

	Mean	Variances	MAD	SNR	MAD
Meta data	0.00324	0.00172	0.02665	—	—
Processed data	0.00261	0.00074	0.01532	110.19721	0.40392

**Table 2:** Statistical characteristics of the data before and after processing.

Model	MSE	RMSE	*R* ^2^	MAPE (%)
LSTM	1.3539	1.1687	0.7973	6.08
LSTM-P	0.9453	1.0069	0.8862	4.81

## Data Availability

The labeled datasets used to support the findings of this study are available from the corresponding author upon request.
